# Effect of Multidisciplinary Team Continuous Nursing on Glucose and Lipid Metabolism, Pregnancy Outcome, and Neonatal Immune Function in Gestational Diabetes Mellitus

**DOI:** 10.1155/2022/7285639

**Published:** 2022-09-08

**Authors:** Shuping Qi, Yanmei Dong

**Affiliations:** ^1^Department of Pediatrics, The Second Children & Women's Healthcare of Jinan City, Jinan, China; ^2^Department of Gynecology, The Second Children & Women's Healthcare of Jinan City, Jinan, China

## Abstract

**Objective:**

To investigate the effect of multidisciplinary team (MDT) continuous nursing on glucose and lipid metabolism, pregnancy outcome, and neonatal immune function in gestational diabetes mellitus (GDM).

**Methods:**

A total of 90 patients with gestational diabetes mellitus (GDM) from January 2018 to December 2019 were recruited and assigned to receive routine care (routine group) or MDT continuous care (study group) according to different nursing methods. Outcome measures included glucose and lipid metabolism, pregnancy outcomes, and neonatal immune function.

**Results:**

There were no significant differences in glucose and lipid metabolism indices and self-rating anxiety scale (SAS) scores, before nursing. After nursing, MDT continuous care resulted in significantly lower levels of fasting blood glucose (FBG), 2 h postprandial blood glucose (2hPBG), glycosylated hemoglobin (HbAlc), triglyceride (TG), and homeostasis model insulin resistance index (HOMA-IR) versus routine care. After nursing, the SAS scores in the two groups were significantly decreased, with lower results in the study group. Patients in the study group showed better compliance than those in the routine group. MDT continuous care was associated with a significantly lower incidence of premature rupture of fetal membranes, cesarean section, premature delivery, macrosomia, and hypoglycemia versus routine nursing. There were no significant differences in immunoglobulin (Ig) A and IgM levels. Patients in the study group showed a higher IgG level and lower CD3, CD4, CD8, and CD4/CD8 levels than those in the routine group.

**Conclusion:**

MDT continuous nursing could effectively regulate glucose and lipid metabolism and improve pregnancy outcomes and neonatal immune function in patients with GDM.

## 1. Introduction

Gestational diabetes mellitus (GDM) refers to impaired glucose tolerance or diabetes that first occurs during pregnancy [1]. According to statistics, the incidence of GDM has increased by 10%-100% worldwide in the past two decades and the incidence is 1%-14% in different countries; the incidence of GDM is 1%-5% in China, which has been on a rise in recent years [2]. The risk factors mainly include advanced age, obesity, parity, ethnicity, physical inactivity, history of macrosomia, family history of type 2 diabetes, and history of GDM [3]. Many clinical studies have demonstrated that GDM is associated with adverse pregnancy outcomes, and women with GDM are at an increased risk of diabetes after pregnancy. It is predicted that 50% of GDM patients will develop diabetes in 22-28 years after pregnancy, resulting in a heavy economic and medical burden to society and family [4, 5]. Traditional treatment methods mainly rely on existing experience and knowledge and are associated with poor treatment outcomes and a high incidence of adverse pregnancy outcomes [6]. Thus, early intervention and improvement of self-management abilities of pregnant women with GDM are of great significance to reduce adverse pregnancy outcomes [7, 8]. The multidisciplinary team (MDT) model refers to a multidisciplinary team composed of clinicians, dietitians, and nurses to provide cross-departmental nursing intervention, resolve nursing issues, and ultimately improve the quality of care [9, 10]. MDT management in China mainly focuses on patients with diabetes, coronary heart disease, and hypertension [11], and it has been reported that specialist nurse-led MDT continuous nursing intervention in out-of-hospital care of elderly diabetic patients could effectively improve the blood glucose control and reduce the incidence of readmission and adverse events [12, 13]. MDT continuous nursing involves four modules, namely, first visit, follow-up visit, one-day clinic, and postpartum. The first visit module includes GDM specialist assessment, formulation of individualized dietary prescription, pregnancy diet, exercise guidance, lifestyle guidance, and pregnancy body mass management. The follow-up visit module includes evaluation of blood glucose self-management, individualized guidance on blood glucose, nutritional assessment, assessment of body mass gain during pregnancy, fetal monitoring, and guidance on glucose-lowering drugs. The one-day clinic module includes blood glucose monitoring, individualized guidance on diet and exercise, guidance on glucose-lowering drugs, and psychological guidance. The postpartum module includes maternal and newborn body mass assessment, postpartum lifestyle guidance, review, guidance on postpartum glucose management, and breastfeeding. However, the application of MDT mode in patients with GDM is marginally explored, so this study was conducted to investigate the effects of MDT continuous care on glucose and lipid metabolism, pregnancy outcomes, and neonatal immune function in gestational diabetes.

## 2. Materials and Methods

### 2.1. General Information

A total of 90 patients with GDM from January 2018 to December 2019 were selected and assigned at a ratio of 1 : 1 to a study group or a routine group according to different nursing methods. There were no significant differences in the general data between the two groups (*P* > 0.05) (Table 1). The research was approved by the Ethics Committee of the Second Children & Women's Healthcare of Jinan City, No. JN2117.

### 2.2. Inclusion and Exclusion Criteria

Inclusion criteria: pregnant women who were diagnosed with GDM as per the 2010 IADPSG diagnostic criteria for gestational diabetes [14], with singleton pregnancy, with clear consciousness to perform normal communication were included.

The diagnostic criteria for hypertensive disorders during pregnancy, excessive amniotic fluid, premature rupture of membranes, postpartum hemorrhage, and fetal macrosomia [2] are as follows. Hypertensive disorders during pregnancy: pregnant women have BP ≥ 140/90 mmHg (mmHg = 0.133 kPa) for the first time during pregnancy, which returns to normal within 12 weeks after delivery, with negative results of urine protein assay. Excessive amniotic fluid: the volume of amniotic fluid in pregnancy exceeds 2000 mL. Premature rupture of fetal membranes: rupture of fetal membranes occurs before delivery. Postpartum hemorrhage: the volume of vaginal bleeding within 24 hours after vaginal delivery exceeds 500 mL or cesarean delivery exceeds 1000 mL. Fetal macrosomia: neonatal birth mass exceeds 4000 g.

Exclusion criteria: patients with underlying diseases such as hypertension and heart disease, with withdrawal of consent, and with severe mental diseases were excluded.

### 2.3. Nursing Methods

The routine group received routine nursing. Routine nursing included regular prenatal care after diagnosis, routine pregnancy guidance and education, assessment of fetal conditions, body mass management, self-monitoring guidance, psychological counseling during pregnancy, and dietary guidance. The fasting blood glucose (FBG), 2-hour postprandial blood glucose (2hPBG), and glycosylated hemoglobin (HbAlc) were measured at 32 and 37 weeks of pregnancy.

The study group received MDT continuous nursing: ① an MDT team composed of endocrinologists, dietitians, mother-infant specialist nurses, midwives, diabetes specialist nurses, psychological specialist nurses, and rehabilitation instructors was established. ② Nursing issues and solutions: nursing issues such as inadequate health knowledge education and poor self-management ability of patients were jointly discussed and analyzed by the MDT members to enhance the compliance and pregnancy outcomes of patients. ③ Health education [15]: the patients were given health education related to GDM to help them understand the disease and enhance treatment compliance. ④ Self-management education was also carried out to enhance patients' awareness of self-care. ⑤ Psychological intervention: psychological counseling was performed to relieve patients' negative emotions and improve treatment compliance. ⑥ Condition monitoring: the blood glucose and related indicators of patients after delivery were closely monitored, and postpartum dietary guidance was provided. Pregnant women with poor blood glucose control were given insulin injections as appropriate. The total daily nutritional intake of pregnant women (≥1500 kcal/d in early pregnancy and ≥1800 kcal/d in late pregnancy) was calculated according to the patient's prepregnancy body mass index. The daily carbohydrate intake was 50-60% of the total intake (≥150 g/d), the fat intake was 25%-30% of the total intake, and the protein intake was l5%-20% of the total intake. Vitamin and minerals were appropriately supplemented, and the daily intake of dietary fiber is controlled at 25-30 g.

### 2.4. Evaluation Criteria

#### 2.4.1. Glucose and Lipid Metabolism Indicators

An AU5800 automatic biochemical analyzer was used to determine the levels of FBG, 2hPBG, HbAlc, fasting insulin (FINS), total cholesterol (TC), triglyceride (TG), low-density lipoprotein cholesterol (LDL-C), and homeostasis model insulin resistance index (HOMA-IR).

#### 2.4.2. Self-Rating Anxiety Scale (SAS) Score

The SAS includes 20 items, with each item being scored as 0-4 points. A score of <50 indicates no anxiety, 50-59 indicates mild anxiety, 60-69 indicates moderate anxiety, and ≥70 indicates severe anxiety.

#### 2.4.3. Compliance

The self-made questionnaire of our hospital was used for compliance assessment. Dietary compliance: patients adhering to the diet for 6 days or more per week were given 4 points, 3 points for 5 days, 2 points for 3-4 days, and 0 points for less than 3 days. Exercise compliance: patients who exercised 5 times or more per week were given 4 points, 3 points for 4 times, 2 points for 3 times, and 0 points for less than 3 times. Blood glucose monitoring compliance: patients who performed blood glucose monitoring 4 times or more per week were given 4 points, 3 points for 3 times, 2 points for 2 times, and 0 points for less than 2 times. A score of ≥3 points indicates good compliance and <3 points indicate poor compliance.

#### 2.4.4. Pregnancy Outcomes

Hyperhydramnios, fetal membrane, cesarean section, neonatal distress, premature delivery, macrosomia, and hypoglycemia were recorded.

#### 2.4.5. Neonatal Immune Function

The levels of immunoglobulin G (IgG), immunoglobulin A (IgA), and immunoglobulin M (IgM) in peripheral blood of neonates were determined using immunoturbidimetry. The levels of CD3, CD4, and CD8 in T cells were determined using flow cytometry, and the CD4/CD8 values were calculated.

#### 2.4.6. Satisfactory Glycemic Control Criteria for Pregnant Women with GDM

The pregnant women had no obvious hunger, with a fasting glucose value of 3.3-5.3 mmol/L, 2-hour postprandial glucose value of 4.4-6.7 mmol/L, and glycated hemoglobin < 5.5%. Venous blood was collected from pregnant women at 32 and 37 weeks of gestation in the outpatient laboratory to determine FBG, HbAlc, and 2hPBG levels. The values of FBG, 2hPBG, and HbAlc that were normal in two tests were considered satisfactory blood glucose control.

### 2.5. Statistical Analysis

SPSS 22.0 software was used for data analyses, and GraphPad Prism 8 was used to plot the graphics. Enumeration data [*n* (%)] and measurement data (mean ± SD) were analyzed by chi-square and *t*-test, respectively. Differences were considered statistically significant at *P* < 0.05.

## 3. Results

### 3.1. Glycolipid Metabolism

There were no significant differences in glucose and lipid metabolism indices before nursing (*P* > 0.05). MDT continuous care resulted in significantly lower levels of FBG, 2hPBG, HbAlc, TG, and HOMA-IR versus routine care (*P* < 0.05) (Table 2).

### 3.2. SAS Score

There were no significant differences in SAS scores before intervention (*P* > 0.05). After nursing, the SAS scores in the two groups were significantly decreased, with lower results in the study group (*P* < 0.05) (Figure 1).

### 3.3. Patient Compliance

According to the results of the questionnaire survey, 31 patients in the routine group had good dietary compliance, 33 had good exercise compliance, and 30 had good blood glucose monitoring compliance; 43 patients in the study group had good dietary compliance, 44 had good exercise compliance, and 42 had good blood glucose monitoring compliance. Patients in the study group showed better compliance than those in the routine group (*P* < 0.05) (Figure 2).

### 3.4. Pregnancy Outcomes

There were 4 cases of conventional polyhydramnios, 9 cases of premature rupture of fetal membrane, 25 cases of cesarean section, 3 cases of fetal distress, 7 cases of premature delivery, 6 cases of macrosomia, and 6 cases of hypoglycemia in the routine group. There were 1 case of polyhydramnios, 2 cases of premature rupture of fetal membrane, 13 cases of cesarean section, 0 cases of fetal distress, 1 case of premature delivery, 1 case of macrosomia, and 1 case of hypoglycemia in the study group. MDT continuous care was associated with a significantly lower incidence of premature rupture of fetal membranes, cesarean section, premature delivery, macrosomia, and hypoglycemia versus routine nursing (*P* < 0.05) (Table 3).

### 3.5. Neonatal Immune Function

There were no significant differences in IgA and IgM levels (*P* > 0.05). Patients in the study group showed a higher IgG level and lower CD3, CD4, CD8, and CD4/CD8 levels than those in the routine group (*P* < 0.05) (Table 4).

## 4. Discussion

Gestational diabetes mellitus (GDM) is a common complication of pregnancy [16], which refers to impaired glucose tolerance or diabetes that first occurs during pregnancy, more frequently in the second and third trimesters of pregnancy. Previous clinical research has demonstrated that GDM is associated with adverse pregnancy outcomes, and women with concurrent GDM are at an increased risk of diabetes after pregnancy [17]. At present, the clinical treatment focuses on blood glucose control and complication prevention [18]. Traditional treatment mainly relies on existing experience and knowledge, and issues in the aspects of diet, psychology, and exercise are mostly handled by experience, resulting in poor treatment outcomes [19]. The MDT [9] is composed of clinicians, dietitians, and nurses to provide cross-departmental nursing intervention, resolve nursing issues, and ultimately improve the quality of care [20]. MDT is patient-centered, guided by the latest medical research results, and relies on a multidisciplinary team to develop the optimal comprehensive treatment plan for a specific disease with standardization, personalization, and continuity. This model enhances effective communication and recognition between medical and nursing care and promotes in-depth learning and exchange of knowledge and techniques of gestational diabetes among various disciplines. In addition, it ensures the integration and communication between the medical and nursing management departments, with collaboration among the clinical group, management group, and quality control group, resulting in a significant improvement in the glycemic and body mass control of pregnant women with GDM. The results of the present study showed that MDT continuous nursing can enhance the effective communication and recognition between medical staff to improve glucose and lipid metabolism control. MDT continuous nursing carries out comprehensive and professional health education, increases the patient's understanding of the disease and the nursing, pays attention to the patient's emotional changes, relieves the patient's concerns to a certain extent, and improves the negative emotions. Tao et al. stated that the IgG level in the blood of newborns of gestational diabetes patients with poor blood glucose control was lower than that of newborns of gestational diabetes patients with good blood glucose control. Combined with the results in the present study, it indicates that MDT continuous care resulted in a superior immune function of newborns and better blood glucose control versus routine care.

## 5. Conclusions

MDT continuous nursing effectively regulates glucose and lipid metabolism in patients with GDM and improves pregnancy outcomes and neonatal immune function, so it is worthy of clinical promotion. The innovation of this study is the use of patient-centered MDT continuous nursing, which relies on a multidisciplinary team to develop an optimal comprehensive treatment plan that is standardized, personalized, and continuous, thereby enhancing the quality of life of patients. However, the limitation of this study lies in the absence of detailed studies on the intelligence and development of the children, which will be investigated in future studies.

## Figures and Tables

**Figure 1:** Comparison of SAS scores before and after nursing. ^∗^*P* < 0.05.

**Figure 2:** Comparison of patient compliance. ^∗^*P* < 0.05.

**Table 1:** Comparison of general data ($\bar{x}\pm s$).

Group (*n* = 45)	Age	Epilepsy	Parity	Prepregnancy BMI	Body mass
Conventional group	28.17 ± 4.03	38.52 ± 1.08	1.41 ± 0.42	24.01 ± 2.95	63.88 ± 8.25
Study group	28.54 ± 3.83	38.65 ± 1.11	1.52 ± 0.39	23.86 ± 3.14	64.12 ± 7.98
*T*	0.446	0.563	1.287	0.234	0.140
*P*	0.657	0.575	0.201	0.816	0.889

**Table 2:** Comparison of glucose and lipid metabolism parameters before and after nursing intervention between the two groups ($\bar{x}\pm s$).

Group (*n* = 45)	Time	FBG (mmol/L)	2hPBG (mmol/L)	HbAlc (%)	FINS (mmol/L)
Conventional group	Preintervention	7.81 ± 1.52	10.56 ± 2.48	6.51 ± 1.24	11.22 ± 2.85
	Postintervention	6.46 ± 1.53^∗^	7.94 ± 2.41^∗^	5.82 ± 1.61^∗^	11.42 ± 2.73
Study group	Preintervention	7.91 ± 1.61	10.58 ± 2.43	6.58 ± 1.12	11.29 ± 2.38
	Postintervention	5.63 ± 1.28^∗^	7.01 ± 1.98^∗^	5.13 ± 1.13^∗^	11.52 ± 3.31
*T*	—	0.303/2.791	0.039/1.904	0.281/2.353	0.126/0.156
*P*	—	0.763/0.006	0.969/0.049	0.779/0.021	0.900/0.876
Group (*n* = 45)	Time	TC (mmol/L)	TG (mmol/L)	LDL-C (mmol/L)	HOMA-IR
Conventional group	Preintervention	5.63 ± 0.88	2.81 ± 0.73	3.19 ± 0.88	1.65 ± 0.44
	Postintervention	4.83 ± 0.68	2.43 ± 0.54^∗^	3.11 ± 0.69	1.31 ± 0.35^∗^
Study group	Preintervention	5.71 ± 0.84	2.82 ± 0.81	3.17 ± 0.91	1.64 ± 0.45
	Postintervention	4.78 ± 0.71	2.21 ± 0.46^∗^	3.02 ± 0.68	1.02 ± 0.23^∗^
*T*	—	0.441/0.341	0.062/2.080	0.106/0.623	0.107/4.645
*P*	—	0.660/0.734	0.951/0.040	0.916/0.535	0.915/<0.001

Note: *T* value and *P* are the comparison results before and after nursing. ^∗^*P* < 0.05.

**Table 3:** Comparison of pregnancy outcomes (%).

Group (*n* = 45)	Hyperhydramnios	Fetal membrane	Cesarean section	Fetal distress	Premature	Macrosomia	Hypoglycemia
Conventional group	4 (8.89)	9 (20.00)	25 (55.56)	3 (6.67)	7 (15.55)	6 (13.34)	6 (13.34)
Study group	1 (2.23)	2 (4.45)	13 (26.67)	0 (0.00)	1 (2.23)	1 (2.23)	1 (2.23)
*X* ^2^	1.901	5.075	6.559	3.102	4.939	3.873	3.873
*P*	0.167	0.024	0.010	0.078	0.026	0.049	0.049

**(a):** 

Group (*n* = 45)	Immunoglobulins (g/L)		
	IgG	IgA	IgM
Conventional group	9.36 ± 2.01	0.31 ± 0.08	0.17 ± 0.07
Study group	10.38 ± 2.62	0.28 ± 0.09	0.16 ± 0.08
*T*	2.072	1.671	0.631
*P*	0.041	0.098	0.530

**(b):** 

Group (*n* = 45)	T cells (%)			
	CD3^∗^	CD4^∗^	CD8	CD4^∗^/CD8^∗^
Conventional group	42.37 ± 9.29	26.98 ± 7.23	25.41 ± 6.04	1.13 ± 0.26
Study group	37.54 ± 8.21	24.17 ± 6.08	23.01 ± 5.16	0.95 ± 0.22
*T*	2.613	2.004	2.027	3.545
*P*	0.011	0.048	0.046	0.001

## Data Availability

The datasets used during the present study are available from the corresponding author upon reasonable request.
